# Realization of English Instructional Resources Clusters Reconstruction System Using the Machine Learning Model

**DOI:** 10.1155/2022/2838935

**Published:** 2022-07-09

**Authors:** Xiaohui Li

**Affiliations:** School of Foreign Languages, Xuchang University, Xuchang 461000, China

## Abstract

Based on ML algorithm, this paper puts forward a method that can search instructional resources through keyword indexing technology, and then cluster and recombine the related results and present them centrally. In this paper, the semantic processing of user query based on the subject index of educational resources is adopted to make up for the deficiency of query semantics, solve the problem of mismatch between query words and document words, and improve the recall and precision of resource retrieval. It is proposed to select the category feature items manually and establish the category feature model. In the environment of small sample set, the weight of category feature items is trained by ML method. The research shows that the user rating of this system is ideal, reaching 93.21% at the highest. In addition, the stability of the system can still reach 89.31% under the condition of relatively large usage, and its performance is excellent. This system can effectively solve the problem of scattered distribution of English instructional resources and make the presentation of knowledge more in line with the needs of users, thereby further improving the utilization rate of English instructional resources and users' satisfaction.

## 1. Introduction

With the advancement of information technology and the continuous advancement of modern educational technology, network communication technology and multimedia technology have developed at an unprecedented rate and have become fully integrated into educational technology development. Modern teaching methods are being adopted by an increasing number of colleges and universities [1]. On the basis of the original campus network, all colleges and universities have established instructional resource management systems to facilitate resource sharing. English is a very practical subject that is closely linked to everyday life. The quality and quantity of learners' language input and output determine the effectiveness of English learning. English instructional resources primarily refer to teaching or learning materials that can assist teachers and students in making better use of teaching and learning data. However, the in-depth development of the construction process has resulted in a slew of issues. On the one hand, due to the rapid growth in the number of instructional resources, users must devote a significant amount of time to obtaining their own English instructional resources from the vast resources available. However, as the number and types of English instructional resources grow, the instructional resource database is no longer a simple database capable of storage and management, and the original centralized management of resources is unable to meet the needs of practical application. As a result, research into instructional resource management is required. In the fields of online education and artificial intelligence [2, 3], the service of instructional resources is gradually becoming an important research topic and hot spot, attracting the attention of more and more researchers. The traditional classification system of teaching network resources lacks logicality and standardization, and it cannot reveal the logical relationship between resources. English teaching network resources are multidimensional, dynamic, and interactive. Due to the growing number of instructional resources, users must devote a significant amount of time to effective retrieval. At the same time, this paper investigates the clustering reconstruction of instructional resources in order to maximize the utilization efficiency of instructional resources.

ML (machine learning) [4–6] is a sub-field of computer science. It started with the research of pattern recognition [7] and computational learning theory, and then entered the field of artificial intelligence. Study the data learning and prediction algorithm of ML, build a model from sample input, and make predictions or decisions through data driving. Learning in ML can be divided into three categories: supervised learning, unsupervised learning, and reinforcement learning. In ML, common classification algorithms include naive Bayes, support vector machine, K nearest neighbor, decision tree, neural network, etc. In the process of clustering, there is no need to mark the data, but the result of clustering is to find out the internal structure and representation of the data. Clustering [8, 9] itself is not an automatic task, but an iterative process of interactive multi-objective optimization. Usually, data preprocessing and model parameters need to be modified until the results reach the required attributes. And common clustering algorithms include partition method, hierarchical method, density-based method, grid-based method, and model-based method. This paper studies the clustering reconstruction of English instructional resources based on ML algorithm. The innovations of the article are as follows:

1. In this paper, ML algorithm is systematically applied to realize the clustering reconstruction of instructional resources, and on the basis of it, efficient resource retrieval service is provided for users. According to the organization mode of the full-text index database of educational resources and the user query structure after semantic processing, the system automatically generates the retrieval scheme. This paper puts forward the process of educational resource retrieval and the correlation ranking algorithm, so as to obtain efficient retrieval performance and ensure that the retrieved resource documents can meet the user's query requirements. At the same time, the calculation method of the matching degree between English instructional resources and category feature models is given.
2. The model of this paper adopts the solution of twice indexing classification storage model, which establishes a reverse index table in the traditional calculation results and classifies the instructional resources by weight in the second calculation. In this way, after two classifications, the index is a directional index table and a reverse index table with weights. At the same time, aiming at the shortcomings of the traditional retrieval methods of educational resources, this paper puts forward a method of expressing users' query requirements by using query outline. The research shows that this system can effectively solve the problem of scattered distribution of English instructional resources and make the presentation of knowledge more in line with the needs of users, so as to improve the effective utilization rate of English education resources.

## 2. Related Work

Lantada et al. applied the clustering algorithm to the resource classification and retrieval in the instructional resource management system, designed and implemented an instructional resource management system based on the clustering algorithm, and verified the availability of the system through tests [10]. On the basis of the teaching reference book system, Shang proposed a clustering retrieval system of characteristic words of instructional resources [11]. The system adopts the technology combining traditional retrieval and feature word clustering to realize the reorganization of instructional resources. Jiang and Li pointed out that the current instructional resource management system in the campus network environment is mainly composed of multimedia cluster servers scattered in grid nodes. The resource scheduling server in the grid system uniformly allocates and uses all resources to achieve effective aggregation and sharing of computing resources, data resources, and service resources [12]. Ko et al. discussed the classification method of teaching network resources, studied how to use the method of combining manual and ML to establish the category feature model, and briefly described the basic idea of the K nearest neighbor classification method [13]. Oku and Sato applied the emerging storage model-cloud storage to the integration of online education resources, thus building an “education cloud.” In this way, the full sharing of instructional resources can be achieved, the construction cost of the distance education system can be reduced, and the storage management of network instructional resources can be standardized [14]. Chen mainly analyzes and studies the current demand for instructional resource storage in colleges and universities and the storage model of massive instructional resources. According to the existing experimental conditions of a school, a fully distributed Hadoop cluster was built and deployed and the storage model was tested [15]. Do et al. proposed a word2vec-based clustering method to achieve clustering, which can narrow the search range, improve efficiency, and make user positioning more accurate [16]. Gholaminejad and Anani Sarab studied the key issues of students' cognitive ability diagnosis in instructional resource recommendation and using ML technology to improve the recommendation accuracy, and proposed an instructional resource recommendation algorithm based on the CUPMF model [17]. This method can push the instructional resources that match the learning level to the student users in a targeted manner according to the student users' learning goals, cognitive ability level, and other personality characteristics. Based on the curriculum resource theory, Hawrylak et al. explored the development of English curriculum resources and their use in English teaching from a practical perspective [18]. Blair et al. designed a reasonable retrieval resource fusion scheme based on the structure of the query outline. It realizes one-click educational resource retrieval through user query decomposition, query semantic processing, educational resource retrieval, retrieval resource screening, relevant content extraction, and retrieval content integration; it can quickly generate the required teaching content according to user queries, which is convenient for users [19].

This paper makes an in-depth analysis and discussion of relevant literature, and then studies the realization of clustering and reconstruction system of English instructional resources based on ML algorithm. Aiming at the problems of scattered distribution of instructional resources and time-consuming retrieval, this paper puts forward some solutions. The method proposed in this paper can search the instructional resources by keyword indexing technology, and then cluster and recombine the related results and present them centrally. At the same time, the experiment shows that the educational resource retrieval method proposed in this paper can well support the information retrieval and clustering reorganization of multi-source educational resource database and quickly generate various teaching contents required by users.

## 3. Methodology

### 3.1. Utilization of English Instructional Resources

The rapid development of network technology and multimedia technology has brought new opportunities for the development of education. The close combination of computer processing technology and educational technology has greatly promoted the pace of educational informatization. English is a highly practical subject closely related to life. The efficiency of English learning depends on the quality and quantity of learners' language input and output. The development and utilization of rich and diverse curriculum resources can ensure the quality and quantity of students' language input, create conditions for students to study selectively according to their own learning needs and the most suitable learning channels, and provide a vibrant source for English teaching [20]. Generally speaking, instructional resources refer to all elements of teaching in the teaching process, which mainly include information data to support teaching and funds, materials, information, and so on in teaching and serving teaching. In a narrow sense, instructional resources mainly include teaching materials, teaching environment and teaching support system. Information instructional resources have the following characteristics: (1) digitization of instructional resources; (2) mass storage; (3) intelligent management; (4) multimedia display; (5) it has certain interactivity. English curriculum is rich in curriculum resources, and actively developing and rationally utilizing curriculum resources is an important part of English curriculum implementation. It embodies the spirit of curriculum reform, meets the needs of English teaching, and is of great significance for changing students' learning style and promoting teachers' professional growth. The types of English educational resources mainly include the supporting educational materials of teaching materials, such as audio and video, pictures, question bank, test papers, and lesson plans. Usually, the school will create an effective instructional resource platform for a large amount of multimedia information and data. In this way, the data management will be established, which will not only help students acquire knowledge, but also enrich and broaden their knowledge and horizons to a greater extent.

According to their sources, educational resources can be divided into two categories: one is the resources uploaded by users who are mainly school teachers through this platform; the other is the shared resources provided by third-party partners such as schools, educational management institutions, and publishers of teaching materials. English teaching emphasizes learners' individualized learning. As students' learning needs are different, and their learning styles and strategies are different, a single learning resource and learning channel cannot meet students' learning needs, and it is not conducive to giving full play to their respective potentials [21]. The specific classification of instructional resources is as follows: (1) media resources: animation, text resources, video resources, image resources, and audio resources; (2) test question bank: the test question bank is based on the relevant education situation, the information of test questions is collected together in the form of computer, and the whole set of electronic test questions constitutes the test question bank; (3) electronic test paper; (4) answers to frequently asked questions; (5) teaching courseware and network courseware; (6) resource index: some index resources set for detecting instructional resources; (7) online courses. In fact, online educational resources are self-communication of educational resources with the help of online means, so as to maximize the autonomy of learning users. According to the characteristics of educational information resources, relevant personnel use various technical methods and tools to process and sort out instructional resources, which is conducive to the storage, dissemination, retrieval, and utilization of educational information, so as to meet people's demand for information education. Among the information-based instructional resources, those instructional resources that support autonomous learning usually have rich graphics and are transmitted through man-machine interaction. These instructional resources can help students choose what they want to learn and what they are interested in. The model of English instructional resources and the visiting process are shown in Figure 1.

English curriculum resources are rich in content, various in types, and complex in composition. In order to better establish the basic conceptual framework of English curriculum resources and better understand and master them, relevant personnel can distinguish English curriculum resources according to different standards and characteristics. However, due to the multidimensional, dynamic, and interactive characteristics of English teaching network resources, the traditional classification system of teaching network resources lacks logicality and standardization, and cannot reveal the logical relationship between resources. At the same time, the traditional search technology is generally based on keyword search, but in large-scale online education applications, it is difficult to quickly find the teaching content users need by using keyword search for educational resources, and the efficiency is extremely low. To some extent, this restricts the development of English instructional resources system and reduces the utilization rate of English instructional resources. With the rapid development of educational informatization, it is very necessary to formulate a set of reasonable management and use scheme of educational resource pool in view of the large amount of multi-source unstructured educational resources on the integrated learning cloud platform. At present, the instructional resource database is no longer a simple database capable of storage and management, and the original centralized resource management method cannot meet the needs of practical application. This kind of storage management mode similar to “behind closed doors” also makes the instructional resources lack of sufficient sharing, which leads to the repeated development of resources and a great waste of instructional resources. Based on this, this paper studies the clustering reconstruction of English instructional resources based on ML algorithm.

### 3.2. ML-Based Cluster Reconstruction System of English Instructional Resources

Educational resources come from a wide range of sources with different forms. Common document formats include word, pdf, ppt, etc. Firstly, according to the different document formats, this paper selects the corresponding document parser to process its information. The process of text preprocessing mainly includes three parts: text sentence segmentation, Chinese word segmentation, and stop words filtering. This paper defines the specific knowledge content unit as a paragraph. Although this definition is a little rough, a paragraph unit also contains rich information, and at the same time, different paragraph units also represent mutually independent contents. Therefore, this division still has certain significance. The main server of the system is mainly responsible for the following work: the servers of the sub-nodes distribute new data or request expired inspection and testing center servers; the master server controls the load balancing, garbage collection, and GFS file saving of the system. In addition, it also solves the modification operation in the model stage. Full-text retrieval is the core technology involved in the retrieval of educational resources. It is an information retrieval method that takes all kinds of data as the processing object and realizes according to the content of data resources rather than their external characteristics. Full-text retrieval technology provides convenient data management tools and powerful data query functions, which can help people sort out massive document resources and quickly and conveniently query any information they want. The framework and process of English instructional resource retrieval are shown in Figure 2.

Because the catalogue of instructional resources is stored in the resource scheduling server in the form of text, before clustering, the text data must be converted into numerical data that can be processed by clustering algorithm. This system uses vector space model to convert text data. When a job is submitted, it will be divided into many different computing tasks, which are mainly responsible for the division of tasks, task allocation, and reducer, for scheduling each computing node. It is responsible for monitoring the execution state of nodes at the same time, and the Map node is responsible for synchronous control and is also responsible for some optimization of computing performance. Clustering module: It realizes the functions of retrieval and feature word clustering mentioned above and realizes the interaction with readers through visual interface. On the basis of grammatical analysis, a thesaurus is established, which includes all possible words and their semantic information. For the string to be analyzed, match it with the words in the thesaurus according to certain strategies. If the match is successful, all semantic information of the word will be taken out from the thesaurus, and then semantic analysis will be carried out. If the analysis result is correct, the string is a word.

K-means clustering is a vector quantization method, originally from signal processing, and is a popular method of clustering analysis in data mining. K-means algorithm repeats the iterative process of data object allocation and new cluster center generation until the criterion function converges. The criterion is shown in the formula:

(1) $$\begin{array}{c} E=\sum_{i=1}^{k}\sum_{x\in C_{i}}{\left|x-{\bar{x}}_{i}\right|}^{2}, \end{array}$$

where *x* is the data object in the data set cluster *C*_*i*_, ${\bar{x}}_{i}$ is the calculated mean of the cluster *C*_*i*_, and *E* is the sum of squared errors for all the data objects in the data set. In this paper, the update calculation method of the cluster center in the traditional K-means algorithm is modified as follows:

(2) $$\begin{array}{c} z_{i}=\frac{1/n_{i}\sum_{j=1}^{n_{i}}x_{j}^{\left(w\right)}-z_{i-1}}{2}. \end{array}$$

In this paper, relative word frequency is used as the metric, and its calculation method generally adopts the *tf* − *i*  *df* formula in information retrieval. As shown in formula (3), the relative word frequency is jointly determined by the word frequency *tf* and the inverse document frequency *i*  *df*, and the weight *w*_*t*_ of the word item *t* in the document *d* is

(3) $$\begin{array}{c} w_{t}=tf_{t}\times idf_{t}=tf_{t}\times \left(\log\frac{n}{n_{t}}+1\right). \end{array}$$

Document relevance can be measured by the idea of vector space model, and the relevance can be defined by calculating the cosine of the included angle between the subject text vectors of two documents. The calculation formula is as follows:

(4) $$\begin{array}{c} Sim\left(d_{i},d_{j}\right)=\frac{P_{i}\cdot P_{j}}{\left\|P_{i}\right\|\left\|P_{j}\right\|}=\frac{\sum_{k=1}^{n}p_{ik}\times p_{jk}}{\sqrt{\sum_{k=1}^{n}{\left(p_{ik}\right)}^{2}}\times \sqrt{\sum_{k=1}^{n}{\left(p_{jk}\right)}^{2}}}. \end{array}$$

The bottom-up hierarchical clustering method takes each object itself as a class at first and then aggregates these classes into a larger class until all objects are in a class or meet certain termination conditions. In order to obtain more accurate retrieval results, this paper improves the algorithm. The improved scoring algorithm is as follows:

(5) $$\begin{array}{c} \text{Score}\left(q,d\right)=\text{coord}\left(q,d\right)\times \text{queryNorm}\left(q\right)\times \sum_{t^{*}inq}\left(tf\left(t^{*}\right)\times idf\;{\left(t^{*}\right)}^{2}\times norm\left(t,d\right)\right), \end{array}$$

wherein *t*^*∗*^ represents an expanded query keyword set corresponding to the original query keyword *t*. *i*  *df*(*t*^*∗*^) is the inverse document frequency of the extended query keyword set *t*^*∗*^, and its formula can be expressed as follows:

(6) $$\begin{array}{c} idf\left(t^{*}\right)=\log\frac{N}{n_{t^{*}}}+1, \end{array}$$

The method based on statistics is adopted; that is, the index words are determined based on the word frequency *tf*, the inverted word frequency *i*  *df*, and the paragraph length *w*. The formula is

(7) $$\begin{array}{c} d_{i}=\frac{tf\times idf}{w},\\ w=\sqrt{w_{1}^{2}+w_{2}^{2}+w_{3}^{2}+\ldots ,+w_{n}^{2}}, \end{array}$$

where *w*_*i*_ is the *i* th word in the resource *tf* × *i*  *df*. In order to be able to determine the final feature word, the system will set a threshold; that is, when the *d* is greater than the threshold, it will be regarded as a feature keyword. The recall and precision ratios can be expressed by formulas as follows:

(8) $$\begin{array}{c} \text{Recall}=\frac{\left|R_{a}\right|}{\left|R\right|},\\ \text{Precision}=\frac{\left|R_{a}\right|}{\left|A\right|}. \end{array}$$

Among them, *R* represents the set of all related documents, *A* represents the set of retrieved documents, and *R*_*a*_ represents the set of retrieved related documents.

Grid the data space, then move the data points to the high-density grid according to the density distribution of the data points in the grid, and then search the edge of the contracted grid space, so as to determine each cluster according to the edge grid. After getting the text paragraphs and the corresponding description information, a very important step is to establish the index of these text-based instructional resources. The establishment of index can improve the retrieval efficiency and quickly find the required paragraphs by matching the content of paragraphs with keywords. Massive data processing necessitates the use of a distributed system with ample distributed data storage capacity and strong computing support. Massive amounts of data can be stored using a distributed file system. These files are distributed on each node's local disk, but they maintain logical data independence and connection, and data visitors keep the data files after the execution is complete. The process of dividing similar items in a document set into different clusters is known as clustering in text analysis. Within a cluster, these documents can be thought of as a collection of similar items, but different items between clusters. We can simplify the features that can be processed by performing preliminary data processing. The next step is to find a function that can compare any two data points from two households. After text preprocessing, instructional resources' knowledge content is divided into smaller granularity, and these paragraph units serve as the foundation for knowledge reorganization. The MapReduce computing framework provides several distributed file system data block storage and data management capabilities that can be backed up multiple times in order to provide massive data storage capacity. In this paper, user dictionaries and stop words dictionaries are built to help IK Analyzer's word segmentation tool improve accuracy and lay a good foundation for semantic understanding of subsequent user queries and retrieval of educational resources, with a focus on primary and secondary education.

## 4. Result Analysis and Discussion

This system runs under the Windows operating system, the database is Oracle, and the main programming environment is based on JDK. In addition, the system adopts JSP and Tomcat to realize the visual interface. All kinds of instructional resources are distributed on 5 servers. The client uses Core Duo, clocked at 2.6 GHz and 16 GB of memory. The data set selected in the experiment is Iris data set which is often used for cluster analysis in UCIML data set. The data of the experiment in this chapter are shown in Table 1.

In order to test the specific clustering effect, this chapter tests about 500 educational resources. Because the keyword index clustering method is mainly adopted, the accuracy of each category after a different keyword clustering is mainly evaluated. Firstly, manually evaluate whether the articles in each category after clustering are related to the feature words, and then calculate the percentage of related articles. The system clustering effect is shown in Figure 3.

Retrieval efficiency is the key standard to evaluate the performance of an information retrieval system. The technical standards to measure retrieval efficiency mainly include response time, recall rate, and precision rate. Response time refers to the time that users wait for the results to be returned after inputting query statements, and it is a measure of the time for the retrieval system to respond to users' needs.  Figure 4 shows the retrieval accuracy of different systems.

In this paper, firstly, the digital resources are preprocessed and the corresponding indexes are established. Then, the retrieval results are obtained and clustered according to the user's request. Finally, the clustering results are output and presented to the user. Select 200 users, use different systems, respectively, and then rate the systems. Collect and sort out the user scores, and get the results of user satisfaction scores of different systems as shown in Figure 5.

It can be seen that this system's satisfaction accounts for a significant portion of the user satisfaction scores for various systems. This demonstrates that the system's functions in this paper are more in line with the user's needs, and it can roughly meet the user's system requirements. Two of the most useful indexes in model evaluation are chosen in this paper: precision and recall. The ratio of retrieved related documents to all related documents in the document collection is used to assess a retrieval system's ability to locate all related documents. The ratio of relevant documents retrieved to total documents retrieved is called accuracy, and it is a measure of how well the retrieval system filters out irrelevant documents. With these two indexes, ten experiments were conducted to verify the model's retrieval quality. The experimental results of the two indexes are shown in Table 2.

On the basis of analyzing the model of educational resources, this paper improves the inverted index structure in Lucene index engine in order to improve the retrieval speed of educational resources. In addition, through the subject index of educational resources, users' queries are semantically processed, thus improving the accuracy of educational resources retrieval. The comparison results of operating efficiency of different systems are shown in Figure 6.

Compared with other systems, the running efficiency of this system is higher. This shows that the system in this paper has certain superior performance and meets the initial development requirements of the system. When building a cluster, this paper considers the number of cluster nodes, and at the same time, setting the number of nodes in the cluster to process data has obvious influence on the storage and processing performance of data resources. In the setting process, the relationship between the number of nodes and the file size is comprehensively considered. Comparing the stability test results of different systems, draw a line chart, and the results are shown in Figure 7.

It can be seen that the system in this paper still has certain stability in the case of relatively large usage. This shows that the stability of this system is better. A large number of studies in this chapter show that the user rating of this system is ideal, reaching 93.21% at the highest; in addition, the stability of the system can still reach 89.31% under the condition of relatively large usage, and its performance is excellent. The results show that clustering reconstruction can effectively improve the retrieval efficiency of instructional resources, thus improving the overall performance of instructional resources management system.

## 5. Conclusions

With the rapid advancement of information technology and the continuous advancement of educational informatization construction, all types of instructional resources produced by schools in the process of teaching informatization are rapidly increasing. Traditional methods of storing and retrieving instructional resources have proven insufficient to meet rising demand, leaving schools with serious issues such as dispersed instructional resources, low resource utilization, and high resource maintenance costs. As a result, it is critical to investigate the cluster reconstruction system for English instructional resources, as it has practical implications. Based on this, this paper proposes a method based on a machine learning algorithm that can search instructional resources using keyword indexing technology, cluster and recombine related results, and present them all in one place. At the same time, in order to address the shortcomings of traditional retrieval methods for educational resources, this paper proposes the use of query outline to express users' query requirements. The findings show that this system can effectively address the problem of dispersed distribution of English instructional resources and align knowledge presentation with user needs. To increase the effective use of English educational resources, the user rating for this system is ideal, according to the research, with the highest score being 93.21 percent. Furthermore, even with relatively high usage, the system's stability can still reach 89.31%, and its performance is excellent. This system can effectively increase the rate of use of English instructional resources and user satisfaction, as well as meet the needs of users. Simultaneously, clustering reconstruction can improve the retrieval efficiency of instructional resources, thereby improving the overall performance of the instructional resources management system. This paper provides an overview of the key technologies used in the English instructional resource clustering reconstruction system and has produced some research findings, but there are still some flaws. The weighting of keywords in the expanded query keyword set is not given a standard in this paper. To formulate a more appropriate weight setting standard, more experiments are needed to clarify the impact of setting the weights of query values on retrieval accuracy.

## Figures and Tables

**Figure 1:** English instructional resource model and access process.

**Figure 2:** English instructional resources retrieval framework and process.

**Figure 3:** Cluster effect of system.

**Figure 4:** Retrieval accuracy of different systems.

**Figure 5:** Results of user satisfaction rating of different systems.

**Figure 6:** Comparison of operating efficiency of different systems.

**Figure 7:** Comparison results of stability of different systems.

**Table 1:** Settings of experimental data.

Serial number	Index	Data
1	Number of users	600
2	Number of resources	1428
3	Number of scores	90000 articles
4	Sparse level	94.17%
5	Sub-data set	5

**Table 2:** Experimental data of evaluation indicators.

Number of experiments	Recall ratio	Precision ratio
1	86.15	89.36
2	88.87	88.45
3	88.64	91.34
4	89.18	91.37
5	90.36	91.52
6	89.54	90.84
7	91.32	92.51
8	90.25	90.13
9	89.38	90.34
10	91.15	92.01

## Data Availability

The data used to support the findings of this study are available from the author upon request.
